This article has been retracted.

# The Computer-Aided Design Algorithm of Dyeing and Weaving Graphics from the Perspective of Public Art

**DOI:** 10.1155/2022/2604302

**Published:** 2022-05-25

**Authors:** Yan Cui

**Affiliations:** Fashion Art Design Department, Hubei Academy of Fine Arts, Wuhan, China

## Abstract

With the acceleration of economic development, people put forward higher requirements for clothing style. In this context, the application of traditional patterns has good artistic effects, can show a unique style, and can also express the artistic beauty of clothing through deformation, color distribution, and other forms, and occupies a relatively large position in the design process of dyeing and weaving art. Aiming at the problem of inaccurate extraction of image information from known visual scenes in the original art-aided design, resulting in unclear output images, this paper proposes a computer-aided design algorithm for dyeing and weaving graphics in the field of public art by color segmentation of the known visual scene images according to the set threshold, morphological processing of the segmented images, reducing noise and fractures affecting the acquired connected areas, and formulating extraction rules to screen candidate areas. Furthermore, dense sampling form is used to extract more scale invariant feature transform (SIFT) target features in the candidate area, match the feature points, integrate the coordinate system of known image information into a unified coordinate system, output the design image, and complete the auxiliary design of dyeing and weaving graphics. The results of simulation experiments show that the computer-aided design algorithm of dyeing and weaving graphics in the public art field is more accurate than the original method in extracting information from known images, which helps to solve the problem of clear output dyeing and weaving images, and improves the quality of dyeing and weaving images.

## 1. Introduction

There have been numerous patterns created during the evolution of traditional culture, each with its own unique connotation, which can be seen here. This collection of patterns represents cultural forms from many socioeconomic times and historical contexts, each with its own creative flavor and study significance [1, 2]. At the same time, the art of dyeing and weaving is a widespread textile industry craft that everyone knows about. It is possible to create an environment of traditional beauty by combining traditional designs with dyeing and weaving techniques, which will allow traditional culture to be effectively pass down to future generations. When it comes to utilizing conventional patterns in dyeing and weaving art design, designers must go outside the box in order to create patterns that have personal meaning while also meeting aesthetic design objectives [3–5].

Through the use of appropriate design approaches, dyeing and weaving products can be used to create a diverse and individual ambiance, with the goal of communicating aesthetic beauty. Most of the time, product design is an important link in the dyeing and weaving manufacturing process. If the design effect does not generate a positive creative mood, it will be a damage to the product's future sales. So, the contemporary dyeing and weaving industry is moving in the direction of creative pattern design, and the share of overall design has expanded even higher. Cloth textiles, living bedding, and other textile products, as well as sub-scenarios such as carpets and furniture coverings, are included in the product classification of the dyeing and weaving art industry. With the increasing acceleration of my country's economic progress, people have raised their expectations for dyeing and weaving artworks, which has resulted in higher demand for these types of works. In this setting, designs with traditional Chinese cultural traits have steadily made their way into the realm of dyeing and weaving design, improving the overall level of design and broadening the range of customers. As a result of its distinctive perspective on national style, this pattern style can contribute to the improvement of cultural competitiveness as well as the enhancement of economic benefits. Dyeing and weaving art typically contains pattern material that includes actual item patterns, abstract object patterns, traditional patterns, folk painting patterns, and other types of pattern content. These designs have excellent dyeing and weaving compatibility, and they can transmit a good creative concept through precise characterization, so increasing the overall economic worth of the cloth. Patterns formed on the surface of dyed fabrics can form information with visual effects to convey content and achieve good artistic effects, such as calligraphy fonts, ancient symbolic seals, and ink landscape paintings [6–14]. These patterns have a broad mass base and can be accepted by the general public, can achieve the best design communication goals, and can be beneficial to the economic value of dyed and woven products as well as to the economic value of dyed and woven products [15].

In the field of the art design, software design and hand-painted design are frequently employed. A range of auxiliary design tools and design software that combine functions [1] have emerged as a result of the rapid growth of multimedia technology, which has increased the likelihood of art design being coupled with computer technology. Design of product through sophisticated software platform is becoming increasingly diverse, and its capabilities are becoming increasingly comprehensive which allows designers to polish and evaluate their work on a regular basis. Likewise, it is cost effective as compared to the manual design where we need to buy the software once and then use it simultaneously. The production of design samples using two-dimensional drawing software and three-dimensional model design software, on the other hand, enriches the creativity of visual effects, allows the designer to better present his or her design concepts and innovative ideas, changes the original form of artistic design, and improves the overall quality of the design. It has resulted in seismic shifts in the field of traditional art design and architecture [16–23].

Scene visual understanding is one of the most widely utilized computer technologies in the field of the art design, and it is one of the most widely integrated computer technologies in the field of art design [24, 25]. Aiming to replace the human eye and brain with computers, scene vision understanding is the process of using computers to simulate the visual function of the human eye and brain to perceive, recognize, and understand three-dimensional scenes and objects in the objective world, as well as to analyze complex objects in scene images by integrating with natural language. We design and extract scene information data by identifying distribution problems and describing the collected information as accurately as possible in an appropriate way. It has been demonstrated that using the art-aided design method in conjunction with the visual scene understanding algorithm can help designers in artistic creation to effectively solve the problem of unclear output images caused by inaccurate extraction of scene image information data from images of scenes. As a result, a suitable scene visual understanding algorithm is proposed, which is based on the application background of computer-aided design (CAD) [26–31].

To address the issue of inaccurate extraction of image information from known visual scenes in the original art-aided design, which results in ambiguous output images, this paper proposes a computer-aided design algorithm for dyeing and weaving graphics in the field of public art with the goal of improving accuracy and clarity. By morphologically processing the segmented images, minimizing noise and fractures, influencing the obtained connected areas, and devising extraction procedures to filter potential areas, color segmentation of known visual scene images according to the given threshold can be accomplished. Dense sampling is used to extract more SIFT target features from the candidate area, match the feature points, combine the coordinate system of known picture information into a unified coordinate system, output the design image, and finish the auxiliary graphic design for dyeing and weaving.

The remaining paper is organized as follows.

In subsequent section, application forms of traditional patterns in dyeing and weaving art design is presented along with highlighting various issues associated with these approaches. In Section 3, the proposed computer-aided design methodology is described in detailed by explaining various sections and subsections of the proposed model. Additionally, this article describes in detail how to use these tools to perform specific tasks and achieve goals. Simulation results of the proposed and existing approaches are presented in Section 4. Finally, concluding remarks are given.

## 2. Application Forms of Traditional Patterns in Dyeing and Weaving Art Design

Through the technique of applying traditional patterns, dyeing and weaving art design primarily consists of basic planning carried out through three types of application, namely aesthetics, color, and the development of an environment (or atmosphere creation). Typically, the pattern is tasked with meeting the fundamental needs of the general public, making it necessary to employ a variety of schemes in order to enhance the visual effect, improve the overall performance quality of the overall elements, and enable people to obtain psychological satisfaction during the application process. During the process of creating a dyeing and weaving art design, it is necessary to thoroughly research the content of aesthetics, color, and atmosphere creation, as well as to take effective measures to thoroughly combine traditional patterns with the dyeing and weaving art design in order to achieve good application results.

### 2.1. Aesthetic Application Form

During the use of traditional patterns for dyeing and weaving art design, designers must pay close attention to the aesthetic effect of the patterns and avoid creating a negative visual experience. First and foremost, a differentiated emotion might be established based on the design state in question. The use of straight pattern design, for example, can provide viewers with an intuitive emotional experience while also enhancing the visual effect of dyeing and weaving artworks. The curved design may provide viewers with a smooth and silky visual experience, which is helpful to increase the overall impact of colored materials when they are used in their application process. When designing, it is important to consider the overall aesthetic style, improve the appropriate planning to the greatest extent feasible, and minimize difficulties that arise too suddenly in the design process. In the course of putting classic patterns into practice, designers frequently employ distorted patterns. Following the completion of the relevant stages, it is required to extract the most representational and visually appealing elements, which can then be further optimized and enhanced in order to accomplish good aesthetic goals while also increasing economic benefits. Plant patterns from the past can be employed to further enhance the overall characteristic effect and to achieve the goal of merging culture and beauty during the application design process. For example, the design of the dyeing and weaving of bedding needs to be optimized and reorganized in conjunction with a large number of traditional element patterns in order to produce a certain level of uniqueness, further enhance the user's good experience, and create an overall uniform aesthetic effect.

Designers use traditional patterns in the design process of dyed fabrics in the context of changing modern aesthetic notions. This process allows people to have a positive visual experience while also achieving the goal of passing down traditional culture. Visual cues, repetition and superposition, and other design techniques are all commonly used. Designers can utilize corresponding design methods to increase the beauty of dyeing and weaving art design, as well as to enrich the hierarchy of the overall design, while putting historic patterns into practice. Using traditional patterns with prominent curves, for example, in the process of dying and weaving garment design, designers can incorporate the peculiarities of women's bodies into the visual form, enriching the visual form and enhancing the integration effect of national culture. Designers can utilize brightly colored plants such as peony and lotus in the abdominal and waist areas, and they can create corresponding designs based on the common body characteristics of women to improve the whole design system.

### 2.2. Color Application Form

The use of traditional patterns for dyeing and weaving product design allows designers to better optimize the use of colors so that they can fulfill the criteria of modern aesthetics while also achieving pleasing aesthetic outcomes. As a result of this, a certain degree of cognition will be created by the visual color design, which will further enhance the layering of the overall dyed fabrics, increase the creative expression effect, and is beneficial to the improvement of economic benefits. The primary characteristics of color include hue, purity, and lightness. It is necessary for designers to apply their own color planning capabilities in order to create color design arrangements that conform to the basic positioning and visual qualities of dyed and woven products. There are several advantages to combining conventional patterns and colors, and it can provide depth to a composition by using comparable colors, opposing colors, complementary colors, and other complementary colors, for example. As a result of this procedure, a thoughtful arrangement of color type and filling area as well as other qualities can significantly enhance the visual experience of the spectator and contribute to creating a more overall attractive ambiance.

Traditional patterns are typically made up of colors such as dark red, golden yellow, grass green, and other similar hues. It is possible to achieve a vibrant and good visual impression by using a fair blend of these colors to represent the cheerful environment of colored and woven products. During the application process of conventional designs, cool colors are employed less frequently, and such shades are typically used when a high level of contrast is necessary. Combining blue, black, purple, and other cool colors with warm colors, for example, can boost the decorative impact of the pattern and further enhance the overall visual environment by increasing the contrast between the hues. Furthermore, by rationally matching the applied colors and planning the corresponding space area, it is possible to achieve the effect of expanding the visual space, strengthening the layered sense of the overall dyed and woven products, balancing the viewer's visual space perception, and reducing the likelihood of incongruity problems. Consequently, a good color pattern application form can have substantial effects on people's physical and mental adjustment, which is advantageous to the improvement of the economic worth of dyed and woven products in the marketplace.

### 2.3. Texture Application Form

In the process of designing dyeing and weaving art objects, it is possible to include the texture visual shape of traditional patterns into the final product. This solution is mostly utilized on the surface of carpets, clothing, and other fiber items, and it has the ability to create an abstract aesthetic ambiance through the application of figurative design elements on the surface of these products. The use of large-scale texture visual design can increase the efficiency of design while also increasing the economic benefits. Using the example of a clothing brand, a distinctive texture description effect can be applied to the surface of colored fabrics to serve as geometric rendering, resulting in a strong sense of beauty in the overall fabric, which is favorable to an increase in the value of the overall product. When traditional patterns for dyeing and weaving art design are applied, a reasonable texture application form can further enhance the overall performance effect, allowing the product to have distinct cultural characteristics and high artistic value while also promoting the development of dyeing and weaving as a craft form.

### 2.4. Forms of Atmosphere Creation

People's quality of life has significantly increased as a result of the rapid progress of science and technology in recent years. While this is happening, however, the beautiful art design inside the building has lost some of its original features, which has altered how it is seen and is not favorable to the exchange of emotional connection between individuals. Inside modern structures, cold hues predominate, with fewer decorative patterns and a more straightforward layout of internal utilitarian areas. People's emotional requirements are not taken into consideration, which has a negative impact on the indoor aesthetic atmosphere. As a result, incorporating historic patterns into dyeing and weaving art design in order to create comparable interior decorating can considerably improve the humanized qualities of a structure while also achieving a positive environment creation effect. Traditional pattern decoration has a significant impact on the creation of an interior design atmosphere with humanized qualities when it comes to interior design. People can live and work in a good artistic atmosphere by arranging areas such as bedding, curtains, carpets, and sofa sets to create a soft decorative environment, increase the qualities of humanization and comfort, and live and work in a good creative environment.

Traditional patterns, for example, can be used to represent people's emotional characteristics while also unifying the overall aesthetic style. Dyed fabrics with traditional designs can be used in the construction of interior decorating, and the type of pattern can be chosen according to the designer's desire throughout the construction process. For example, if the residents like a natural-style pastoral ambiance, they can decorate with traditional plant patterns such as peonies, leaves, lotuses, and other such flowers, and use these elements to create a good natural ambiance while still achieving the basic decoration aims. If the residents like a traditional cultural atmosphere, totem components such as dragons and stone lions might be used as decorative elements in the home. Utilizing these arrangements may effectively improve the aesthetic ambiance of interior space, increase the decorative effect of colored fabrics, and be conducive to the ongoing inheritance and development of traditional patterns.

Dyed fabrics can be decorated with traditional designs that have cultural qualities that can be employed in the process of arranging certain places. Using traditional calligraphy fonts, for example, the hotel lobby or tea shop area can be transformed, communicating to guests the meaning of the artist's brushstrokes, thereby accomplishing the goal of preserving national elements and further expanding the communication channels of cultural and artistic charm. Traditional patterns, on the other hand, have a variety of characteristics. In order to create an elegant and noble emotional atmosphere for the hotel, designers can use traditional cultural patterns on-screen dyed fabrics. This will make the overall decoration attractive to the sight and create an elegant and noble emotional atmosphere. It is believed that the eight horses in traditional patterns represent a unique cultural form that can transmit the commercial connotation of success and help to establish a favorable trading environment.

A light atmosphere is created in some antique shops by incorporating blue and white porcelain pieces into traditional designs to further enhance the cultural ambiance of dyed fabrics while also producing a light atmosphere in the business. Furthermore, there is no acknowledgment as a result. Traditional colored and woven clothing, as well as traditional designs, can be a fantastic addition to any wardrobe. As a result, the incorporation of traditional pattern elements into dyeing and weaving art design can result in the creation of a complementary variety. Dyed fabric designers should pay close attention to the corresponding content design, as well as the market environment characteristics of dyed fabrics, in order to maximize the overall visual effect.

## 3. The Proposed Method

In complicated scene photos, the target information or items are obscured by other objects, the color difference changes, and the shape and size of the target information are all changing, making it difficult to extract target information's features from the photographs. As a result, in the art-aided design technique based on the scene visual understanding algorithm, color segmentation of the scene image is conducted first according to the threshold value selected. The effective description area is then morphologically processed in order to produce the candidate area, and the SIFT feature is subsequently utilized to extract the candidate region from the effective description area. We provide the required materials for the integrated design system and screen qualified information to realize art aided design.

Initially, image smoothing procedure is carried out to remove noise which is necessary to smooth up the surface of the fabric before extracting dyeing and weaving patterns from it. In the case of the *F*_0_ norm smoothing filter, the image is smoothed, which means that the intensity of the transition edge is sharpened, the minor intensity jitter is decreased, the major structure is highlighted, and the visible gradient changes are kept. The smoothing of unimportant details is achieved through the deletion of minor non-zero gradients, which helps to emphasize the image's apparent edges. The objective function is calculated based on the input signal *h* and the output signal *k*:

(1) $$\begin{array}{c} \underset{k}{\min}\sum_{q}{\left(k_{q}-h_{q}\right)}^{2}-\alpha e\left(k\right), \end{array}$$

where *e*(*k*) represents the image gradient norm, which is calculated as follows:

(2) $$\begin{array}{c} e\left(k\right)=\#\left\lfloor q\left\|k_{q}-k_{q-1}\right\|\neq 0\right\rfloor . \end{array}$$

Although there are significant differences in the gray values of the stroke pixels and the background pixels of the dyeing and weaving image in some areas, the gray value ranges of the stroke pixels and the background pixels of the dyeing and weaving image will overlap to a certain extent in all areas. In order to make the extraction of strokes easier, the gray value distribution of background pixels should be simplified, and the contrast between the strokes and the background should be effectively stabilized, according to the authors. The original image was therefore subjected to high-frequency lifting filtering using Gaussian blur as the carrier, which was then evaluated. Gaussian low-pass filtering is responsible for the so-called Gaussian blur, and the equation of filter is as follows:

(3) $$\begin{array}{c} L\left(w,v\right)=c^{-\left(dist^{2}\left(w,v\right)/2k^{2}\right)}, \end{array}$$

where dist(*w*, *v*) represents the distance between the origin of the Fourier transform, *k* represents the standard deviation of the Gaussian distribution, which can represent the degree of expansion of the distribution curve.

After being transformed by Fourier, the image has a smooth range of gray levels with the low-frequency components effectively reflecting the overall gray level of the smooth range, and with the high-frequency components effectively reflecting the edge and noise of the image. Using Gaussian blur, you can simplify the specific distribution of gray value of the stroke pixels and background pixels by removing high-frequency components. This can help you ensure that the edge of the stroke is well defined.

We make use of a high-frequency boost filter, then:

(4) $$\begin{array}{c} U_{2}\left(i,j\right)=\min\left[255,U_{0}\left(i,j\right)+△U_{0}\left(i,j\right)\right], \end{array}$$

where *U*_2_(*i*, *j*) represents the output result, *U*_0_(*i*, *j*) represents the grayscale image of the original image, and *U*_1_(*i*, *j*) represents the *U*_0_(*i*, *j*) Gaussian blur result.

Then,

(5) $$\begin{array}{c} △U_{0}\left(i,j\right)=\left\{\begin{array}{cc} 255, & U_{1}\left(i,j\right)=0,\\ \frac{255-U_{1}\left(i,j\right)}{U_{1}\left(i,j\right)}\cdot U_{0}\left(i,j\right), & \text{else.} \end{array}\right) \end{array}$$

ETF is formed, and the ETF formula is optimized based on edge tangential flow, adding high-frequency filtering image gradient amplitude weight function and strengthening the primary contour line features of dyeing and weaving graphics, followed by the following procedures:

(6) $$\begin{array}{c} r\left(i\right)=\frac{1}{f}\sum_{j\in \Omega \left(i\right)}\delta \left(i,j\right)t_{1}\left(j\right)\lambda_{p}\left(i,j\right)\lambda_{n}\left(i,j\right)\lambda_{m}\left(i,j\right)\lambda_{1}\left(i,j\right), \end{array}$$

where Ω(*i*) represents the neighborhood, *λ*_*n*_(*i*, *j*) represents the magnitude weight function, *λ*_*p*_(*i*, *j*) represents the spatial weight function, and *λ*_*m*_(*i*, *j*) represents the direction weight function.

The image gradient vector *t*_0_(*i*) is represented by a vector orthogonal to the image gradient vector during initialization, and then a new high-frequency filter image gradient magnitude weight function, which is as follows:

(7) $$\begin{array}{c} \lambda_{1}\left(i,j\right)=\frac{\left[1+\tan\left(\rho \cdot \chi_{1}\left(j\right)-\chi_{1}\left(i\right)\right)\right]}{2}. \end{array}$$

Anisotropic Gaussian difference filtering is used to extract line maps which are used to improve the overall effect of flow field constructed with the new edge tangential flow field creation. It is known that the FDo *G* filter method has been optimized, and the lines have been improved by high frequency to enhance the characteristics of dyeing and weaving images, the gray image has been replaced by its product *U*_*n*_ as a result of the high-frequency filtering improvement result, and the following steps have been taken:

(8) $$\begin{array}{c} Q\left(d\right)=\int_{-R}^{R}U_{n}\left(l_{d}r\right)\left(H_{\gamma e}r-\beta H_{\gamma d}r\right)gr,\\ U_{n}\left(i,j\right)=\frac{U_{0}\left(i,j\right)\cdot U_{n}\left(i,j\right)}{255}. \end{array}$$

And the variance of *γ*^2^ is

(9) $$\begin{array}{c} H_{\gamma }\left(i\right)=\frac{f^{\left(-i^{2}/2\gamma^{2}\right)}}{\sqrt{2\pi }\gamma }. \end{array}$$

Then, we can conduct the FDo *G*, which is as follows:

(10) $$\begin{array}{c} G\left(i\right)=\int_{-d}^{d}H_{\gamma e}\left(d\right)Q\left(d\right)\text{g}d,\\ G_{1}\left(i\right)=\left\{\begin{array}{cc} 0, & G_{1}\left(i\right)<0;1+\tan G\left(i\right)<\eta ,\\ 1, & \text{else.} \end{array}\right) \end{array}$$

It is intended to use a computer vision algorithm SIFT feature for the feature description of the candidate region of the scene image. SIFT feature, which has the advantages of location information as well as scale signal invariance to the local features of the image, detects and describes the local features of the candidate region while reducing the amount of data that must be processed by the computer. The critical visual information is retained that is required.

The SIFT feature point is typically used as the center of the candidate area in order to increase the amount of sampling and improve the image clarity of the design output. The gradient sum of each pixel in the 1616 window range is calculated in order to make the sampling more sufficient and to improve the image clarity of the output. As illustrated in Figure 1, dense sampling is used in this paper in order to obtain a greater number of SIFT feature points.

To sum up, the flowchart of the algorithm in this paper is shown in Figure 2.

## 4. Simulation Results

This paper is focused on the development of software-enabled patterns linked to dyeing and weaving from the Google Image Library and Baidu Image Library such as forests, mountains, and other natural scenery, lotus, plum, and orchids of plant species, and other patterns connected to dyeing and weaving from other sources. The essential aspects of the relevant graphics are extracted from the collected photographs, and then the dyeing and weaving works that incorporate the important features of the images are created.

This paper takes the common plant lotus in dyeing and weaving as an example, and the proposed algorithm is used to assist in developing the dyeing and weaving pattern based on the lotus image in this paper.  Figure 3 is an image of a lotus flower.

The lotus picture is used to design the dyeing and weaving image in this paper, with the primary color red serving as the background. The dying and weaving diagram, which was assisted by the computer-aided design algorithm of the dyeing and weaving graphics in the public art sector, is shown in Figure 4. The dying and weaving diagram is shown in Figure 4. It can be seen that the computer-aided design algorithm presented in this paper is effective. It is preferable to design the most important aspects of the reference visuals first. Among them, the petals are shown in great detail, and the primary hue is consistent with the surrounding environment. Furthermore, because the primary color is red, the algorithm used in this work automatically ignores the green lotus leaves in the image.

The aided design algorithm described in this study is also contrasted with the classic aided design algorithm. In Reference [25], the design similarity index is used to calculate the measurement index.  Figure 5 depicts a comparison diagram of the two options.

It can be seen that the computer-aided design algorithm of dyeing and weaving graphics in the field of public art is obviously better than the traditional aided design algorithm.

## 5. Conclusion

In the product design process, if traditional patterns are used, then these are very good specifically from the perspective of the artistic effect. These patterns may demonstrate a distinct style and has the capability to convey the aesthetic beauty of clothes through distortion, color distribution, and other forms which are described in literature. These patterns play an essential role in the design process of dyeing and weaving art. However, these patterns have various issues as described above. In this paper, the computer-aided design algorithm for dyeing and weaving graphics is used to successfully extract the image information from existing visual sceneries while also improving the output quality of dyeing and weaving graphics and the visual effect of art-aided design. Simulation results have verified the outstand performance of the proposed scheme.

## Figures and Tables

**Figure 1:** SIFT gradient histogram.

**Figure 2:** Flowchart of our method.

**Figure 3:** Schematic diagram of the lotus dataset.

**Figure 4:** Design-aided lotus dyeing and weaving diagram.

**Figure 5:** Comparison results.

## Data Availability

The data used to support the findings of this study are available from the corresponding author upon request.
